This article has been retracted.

# Expression of Th17/Treg Cells in Peripheral Blood and Related Cytokines of Patients with Ulcerative Colitis of Different Syndrome Types and Correlation with the Disease

**DOI:** 10.1155/2021/4600947

**Published:** 2021-09-23

**Authors:** Jianhua Yu, Shu Wang, Hongsheng Yuan, Tingyue Qiao, Miao Bao

**Affiliations:** ^1^Department of Gastroenterology, Qijiang Hospital, The First Affiliated Hospital of Chongqing Medical University, Chongqing 401420, China; ^2^Chongqing Medical School, Chongqing 401420, China; ^3^Department I of General Surgery, Qijiang Hospital, The First Affiliated Hospital of Chongqing Medical University, Chongqing 401420, China; ^4^Department of Gastroenterology, Yongchuan Hospital Affiliated to Chongqing Medical University, Chongqing 402160, China

## Abstract

**Objective:**

To explore the expression of helper *T* cells 17 (Th17)/regulatory *T* cells (Treg) in peripheral blood and related cytokines of patients with different types of ulcerative colitis (UC) and analyze their correlation with the disease.

**Methods:**

From January 2018 to December 2019, 53 patients diagnosed with UC in our hospital were selected. According to their medical syndromes, they were divided into the damp-heat internal accumulation group (*n* = 35) and the spleen-kidney yang deficiency group (*n* = 18). 21 healthy volunteers were selected as the control group. The Mayo scoring standard was used to determine the severity of the patient's condition. The expression levels of Th17/Treg cells and related cytokines in peripheral blood were compared between the groups. Pearson correlation was used to analyze the correlation between the ratio of Th17 and Treg cells in the peripheral blood of UC patients and the ratio of TH17/Treg with Mayo score.

**Results:**

The peripheral blood Th17 cell ratio and Th17/Treg ratio of the damp-heat internal accumulation and spleen-kidney yang deficiency group were higher than those of the control group; the Treg cell ratio was lower than that of the control group; the peripheral blood Th17 cell ratio and Th17/Treg ratio of the damp-heat internal accumulation group were higher those of the spleen-kidney yang deficiency group; and the proportion of Treg cells was lower than that of the spleen-kidney yang deficiency group (*P* < 0.05). The expression levels of serum IL-6, IL-17, IL-22, and TNF-*α* in the damp-heat internal accumulation and spleen-kidney yang deficiency group were higher than those of the control group; IL-10 and TGF-*β* were lower than those of the control group; the levels of serum IL-6, IL-17, IL-22, and TNF-*α* in the damp-heat internal accumulation group were higher than those of the spleen-kidney yang deficiency group; and both IL-10 and TGF-*β* were lower than those of the spleen-kidney yang deficiency group (*P* < 0.05). The peripheral blood Th17 cell ratio and Th17/Treg ratio in the moderately active period group and severely active period group were higher than those of the lightly active period group; the Treg cell ratio was lower than that of the lightly active period group; the peripheral blood Th17 cell ratio and Th17/Treg ratio in the severely active period group were higher than those in the moderately active period group; and the proportion of Treg cells was lower than that of the moderately active period group. Pearson correlation analysis showed that the proportion of Th17 cells and Th17/Treg in peripheral blood of UC patients were both positively correlated with Mayo score (*r* = 0.762, *r* = 0.777, *P* < 0.001). Treg was negatively correlated with Mayo score (*r* = −0.790, *P* < 0.001).

**Conclusion:**

There are differences in the expression of peripheral blood Th17/Treg cells and related cytokines among UC patients with different syndromes, and the damp-heat content is the most significant. The higher the ratio of Th17 cells in peripheral blood and the degree of Th17/Treg imbalance, the lower the ratio of Treg cells, and the more severe the condition of UC patients, which can provide a preliminary quantitative basis for the TCM classification and severity of the diagnosis of UC.

## 1. Introduction

Ulcerative colitis (UC) is a chronic nonspecific inflammatory disease that mainly affects the rectum and colonic mucosa [1]. Most patients have abdominal pain, diarrhea, Tenesmus, and other clinical features. Both UC and Crohn's disease belong to inflammatory bowel disease [2]. The course of the disease is long and the condition is protracted, sometimes as long as several years or even decades. Its pathology can lead to the involvement of multiple surrounding systems, so it has more complications. Moreover, when chronic inflammation is repeatedly irritated, it also quickly progresses to malignant lesions of the colorectal, which poses a threat to the quality of life and life safety of patients [3]. Regarding the pathogenesis of UC, clinical considerations are mainly about colonic mucosal epithelial cells secreting abnormal mucus glycoproteins, changes in the permeability of intestinal mucosal, and antigens entering the intestinal mucosa, leading to a series of inflammatory changes and immune responses, and further production of inflammatory mediators and antibodies, cytokines, and oxygen free radicals, but its ultimate pathogenesis and reasons still need to be further studied [4–6]. At present, many scholars tend to believe that it may be related to the autoimmune system, among which, *T* helper cell 17 (Th17), regulatory *T* cells (Treg), and cytokines are closely related to their occurrence and recurrence [7]. UC belongs to the category of “diarrhea” in traditional Chinese medicine. In the theory of traditional Chinese medicine syndrome differentiation, the common syndrome types of UC include actual syndrome represented by damp-heat internal accumulation and deficiency syndrome represented by spleen-kidney yang deficiency. In previous studies, there have been many reports on the role of Th17/Treg subgroups in the pathogenesis of UC, and most of them focused on the exploration of western medicine mechanisms. This study explored the differences in Th17/Treg cell and related factor expression in UC patients with different traditional Chinese medicine syndromes and its correlation with the condition of disease, in order to provide a theoretical basis for traditional Chinese medicine syndrome differentiation of UC and provide a basis for clinical treatment. See the following report for details.

## 2. Materials and Methods

### 2.1. General Information

From January 2018 to December 2019, According to their medical syndromes, 53 patients with UC were divided into the damp-heat internal accumulation group (*n* = 35) and the spleen-kidney yang deficiency group (*n* = 18). Another 21 healthy volunteers were selected as the control group. The damp-heat internal accumulation group consisted of 20 males and 15 females. The age ranged from 23 to 59 years, with an average of (35.59 ± 14.26) years. The spleen-kidney yang deficiency group consisted of 10 males and 8 females. The age ranged from 24 to 60 years, with an average of (36.21 ± 13.95) years. The control group consisted of 12 males and 9 females. The age ranged from 20 to 58 years, with an average of (35.65 ± 13.21) years. There was no statistical difference in baseline information between the three groups (*P* > 0.05), comparable.

### 2.2. Inclusion Criteria

(1) It conformed to the relevant Western medicine diagnosis in the “Consensus on the Diagnosis and Treatment of Inflammatory Bowel Disease (2012 Edition).” This meant (i) persistent or recurrent episodes of diarrhea, mucus pus, and blood in the stool with abdominal pain, Tenesmus, and varying degrees of systemic symptoms; (ii) course of the disease was more than 4 w to 6 w; (iii) there might be extraintestinal manifestations of skin, mucous membranes, joints, and so forth; and (iv) colonoscopy was the most important basis for diagnosing UC; under the microscope, it can be seen that the intestinal mucosa often has superficial erosions and ulcers; there are purulent secretions, mucosal congestion, edema, and blurred blood vessel texture; and the lesions appear continuous and diffuse distribution from the rectum. (2) It conformed to the relevant traditional Chinese medicine diagnosis in the “Guidelines for the Diagnosis and Treatment of Ulcerative Colitis Integrated Traditional Chinese and Western Medicine” (2011 edition). Among them, patients with damp-heat internal accumulation syndrome manifested as yellowish complexion or yellowish sclera, dirty mouth, yellow urine, mucus or blood and heavy taste in the stool, white and greasy tongue coating or yellow, and thick and greasy tongue coating. Patients with spleen-kidney yang deficiency syndrome manifested as pale complexion, low speech, anorexia, sore waist and knees, tinnitus, long and clear urine, difficult and hard stool, and blood in the stool. (3) Age was from 18 to 60 years. (4) No intestinal infections in the past 1 month. (5) No antibiotics and probiotics in the past 1 month. (6) The patient and family members agreed and signed the informed consent book.

### 2.3. Exclusion Criteria

(1) Infectious colitis such as ischemic colitis, amoebic dysentery, and bacillary dysentery; (2) serious complications such as intestinal perforation, local stenosis, and intestinal obstruction; (3) patients with severe primary disease and mental illness of the liver, kidney, hematopoietic system, and so forth; (4) patients with a history of malignant tumors; (5) patients with autoimmune diseases or infectious diseases at onset; (6) patients during pregnancy and lactation; and (7) known blood diseases in the past or were using bone marrow suppression and/or stimulating drugs.

### 2.4. Criteria for Elimination and Drop-Off

(1) Patients who could not use standard medications during the observation period; (2) those who lacked cognitive and expressive function of things; and (3) those who could not judge their curative effect during the observation period.

### 2.5. Research Methods

The proportion of Th17 and Treg cells in peripheral blood was detected by flow cytometry; Serum interleukin (IL-6, IL-17, IL-22), tumor necrosis factor-*α* (TNF-*α*), and IL-10, transforming growth factor-*β* (TGF-*β*) levels were detected by enzyme-linked immunosorbent assay. The operation method was in accordance with the kit instructions strictly. The kit was provided by Epison (Shanghai) Biotechnology Co., Ltd.

#### 2.5.1. Evaluation of Severity of Illness

Mayo scoring standard was used clinically to determine the severity of the patient's illness. The Mayo score was mainly based on the number of bowel movements, the degree of blood in the stool, the changes of endoscopic, and the overall evaluation of the physician. Mayo score <2 points was divided into symptom remission period (*n* = 18), 3 to 5 was divided into mild activity period (*n* = 13), 6 to 10 was divided into the moderately active period (*n* = 12), and 11 to 12 was divided into the severely active period (*n* = 10).

### 2.6. Statistical Methods

Use SPSS 22.0 software to process. The measurement data was expressed as ($\bar{x}$ ± *s*), analysis of variance was used for multigroup comparison, and *t*-test was used for pairwise comparison. Pearson correlation was used for correlation analysis. The count data was expressed as a rate (%), and *χ*^2^ test analysis was used for comparison. *P* < 0.05 indicated that the difference was statistically significant.

## 3. Results

### 3.1. Comparison of Th17 and Treg Cell Ratios and Th17/Treg Ratios in Peripheral Blood of Different Groups

The peripheral blood Th17 cell ratio and Th17/Treg ratio of the damp-heat internal accumulation group and the spleen-kidney yang deficiency syndrome group were higher than those of the control group; Treg cell ratio was lower than that of the control group; peripheral blood Th17 cell ratio and Th17/Treg ratio of the damp-heat internal accumulation group were higher than those of the spleen-kidney yang deficiency group; and the proportion of Treg cells was lower than that of the spleen-kidney yang deficiency group (*P* < 0.05), as seen in Figure 1.

### 3.2. Levels in Different Groups Comparison of Serum-Related Cytokine Expression

The expression levels of serum IL-6, IL-17, IL-22, and TNF-*α* in the damp-heat internal accumulation and spleen-kidney yang deficiency group were higher than those of the control group; IL-10 and TGF-*β* were lower than those of the control group; the levels of serum IL-6, IL-17, IL-22, and TNF-*α* in the damp-heat internal accumulation group were higher than those of the spleen-kidney yang deficiency group; and both IL-10 and TGF-*β* were lower than those of the spleen-kidney yang deficiency group (*P* < 0.05), as seen in Figures 2 and 3.

### 3.3. Comparison of the Ratio of Th17 and Treg Cells and Th17/Treg Ratio in Peripheral Blood between the Active UC Groups

The peripheral blood Th17 cell ratio and Th17/Treg ratio in the moderate and severe active phase group were higher than those of the lightly active phase group; the Treg cell ratio was lower than that of the lightly active phase group; the peripheral blood Th17 cell ratio and Th17/Treg ratio in the severely active phase group were higher than those in the moderately active group; and the proportion of Treg cells was lower than that of the moderately active group (*P* < 0.05), as seen in Figure 4.

### 3.4. The Relationship between the Proportion of Th17, Treg Cells in the Peripheral Blood and the Ratio of Th17/Treg and the Condition of UC Patients

Pearson correlation analysis showed that the proportions of Th17 cells and Th17/Treg in peripheral blood of UC patients were both positively correlated with Mayo score (*r* = 0.762, *r* = 0.777, *P* < 0.001). Treg was negatively correlated with Mayo score (*r* = −0.790, *P* < 0.001), as seen in Figure 5.

## 4. Discussion

UC is currently one of the more difficult diseases in the treatment of gastroenterology, which is mostly related to multiple factors such as genetic susceptibility, intestinal mucosal immunity, environment, and intestinal microbes [8, 9]. In Chinese medicine syndrome differentiation, UC is caused by the combined action of original deficiency and superficial reality. From the surface symptoms, the patient started the disease because of the invasion of dampness, but at the root, the patient started the disease because of the weakness of the spleen. Based on this, UC can be divided into six syndrome types. Among them, the actual syndrome includes the syndrome of damp-heat internal accumulation and the syndrome of qi-blood stasis; the deficiency syndrome includes the syndrome of spleen-stomach deficiency and the syndrome of spleen-kidney yang deficiency; and the syndrome of deficiency and actual inclusions is the syndrome of liver depression and spleen deficiency. Evaluating the TCM syndrome types of UC based on relevant clinical indicators and enriching the specific content of TCM syndrome differentiation is of great significance to the TCM treatment of the disease.

The intestinal mucosal immune system is one of the important mechanisms for maintaining the homeostasis of the intestinal mucosal environment. CD4^+^*T* cells are an indispensable and important part of it. Th17 and Treg cells are different cell subdivisions differentiated by CD4^+^*T* cells under the stimulation of different antigens [10, 11]. In recent years, many studies have shown that the imbalance of Th17/Treg in peripheral blood is closely related to the onset of UC. Peripheral blood Th17 cells are helper *T* cells differentiated from CD4^+^*T* cells, which are closely related to human autoimmune diseases [12]. The IL-6 secreted by it is a pleiotropic cytokine with a wide range of effects, which can be rapidly produced in the case of acute inflammation such as tumors, trauma, infection, and stress [13]; IL-17 secreted by it is a key cytokine that induces inflammation and participates in Inflammation occurrence, leading to the occurrence of UC [14]; IL-22 secreted by it is a cytokine attributed to IL-10, which has a dual role of promoting and resisting inflammation and plays an important role in the pathogenesis of UC [15]; and TNF-*α* secreted by it is systemic inflammatory cell factors that mediate the pathological damage of certain autoimmune diseases [16]. Peripheral blood Treg cells are a type of CD4^+^*T* cell subgroup with immunomodulatory function, contrary to the inflammatory effect of Th17 cells; they have the effect of resisting inflammation [17]. Treg cells inhibit intestinal inflammation by secreting anti-inflammatory factors IL-10 and TGF-*β* [18]. Th17 cells and Treg cells work together to maintain the balance of immune function in the body, under normal physiology, the Th17/Treg ratio is in a balanced state, and the Th17/Treg ratio is unbalanced, which can cause the occurrence of UC [19].

The results of this study showed that the Th17 cell ratio and Th17/Treg ratio of peripheral blood in the damp-heat internal accumulation group and the spleen-kidney yang deficiency group were higher than those in the control group; the ratio of Treg cells was lower than that in the control group; the ratio of Th17 cells and Th17/Treg ratio of peripheral blood in the damp-heat internal accumulation group was higher than that of spleen-kidney yang deficiency group; and the ratio of Treg cells was lower than that in the spleen-kidney yang deficiency group. The reason is that the increase of Th17 cells in peripheral blood and the imbalance of Th17/Treg caused by the decrease of Treg cells play an important role in the pathogenesis of UC. Damp-heat internal accumulation is more common in patients with active phases, Th17 cells are inflammatory cells that are mediated by cytokines, when Th17 cells are hyperactive, the secretion of inflammatory factors is increased, thereby aggravating the inflammatory response [20]. The decrease in the number of Tregs and the decreased function reduce the secretion of various anti-inflammatory factors such as IL-10, so it cannot inhibit inflammation and maintain the body's immune balance [21]. Deficiency of yang of the spleen and kidney is more common in the remission period, the number of Tregs is not significantly reduced, which plays a negative regulatory role to a certain extent, but the patient still has an abnormal immune function, which is specifically manifested in the expression level of Th17 and related cytokines in peripheral blood are still higher than those of healthy people. In this study, the expression levels of peripheral blood serum IL-6, IL-17, IL-22, and TNF-*α* in the damp-heat internal accumulation group and the spleen and kidney yang deficiency group were higher than those in the control group; IL-10 and TGF-*β* were lower than those in the control group; the serum IL-6, IL-17, IL-22, and TNF-*α* in the damp-heat internal accumulation group were higher than those in the spleen-kidney yang deficiency group; and the serum IL-10 and TGF-*β* in the damp-heat internal accumulation group were lower than those in the spleen-kidney yang deficiency group. The above results are consistent with the conclusion.

This study showed that the ratios of Th17 cells and Th17/Treg in the peripheral blood of UC patients were positively correlated with the condition, and the ratio of Treg cells was negatively correlated with the condition. In this result, the ratio of Th17 cells and the Th17/Treg ratio increased in the peripheral blood, the ratio of Treg cells decreased in patients with severe UC, the ratios of Th17 cells and Th17/Treg ratio in peripheral blood were positively correlated with Mayo score, and the ratio of Treg cells was negatively correlated with Mayo score. This shows that the proportion of Th17 and Treg cells and their balance are related to the severity of UC, which can be used as one of its evaluation indicators. Therefore, regulating the balance of Th17/Treg cells is a new idea for the clinical treatment of UC.

In summary, there are differences in the expression of peripheral blood Th17/Treg cells and related cytokines among UC patients with different syndromes, and the damp-heat content is the most significant. The higher the ratio of Th17 cells in peripheral blood and the degree of Th17/Treg imbalance, the lower the ratio of Treg cells and the more severe the condition of UC patients. This study can provide a preliminary quantitative basis for the diagnosis of TCM classification and severity of UC, but there are still shortcomings. For example, the sample size is too small and the specific mechanism of Th17/Treg imbalance needs to be further studied and explored.

## Figures and Tables

**Figure 1:** Comparison of Th17 and Treg cell ratios and Th17/Treg ratio in peripheral blood of different groups ($\bar{x}$ ± *s*). (a) Th17 and Treg cell ratios and (b) Th17/Treg ratio. Among them, the ratios of the Th17 cells in the control group, the damp-heat internal accumulation group, and the spleen-kidney yang deficiency group were (3.52 ± 0.54)%, (8.98 ± 1.75)%, (7.25 ± 1.66)%, respectively; the ratios of the Treg cells were (1.28 ± 0.69)%, (0.86 ± 0.33)%, (1.03 ± 0.52)%, respectively; the Th17/Treg ratios were (4.45 ± 1.21), (10.75 ± 2.81), (9.02 ± 2.77), respectively. ^*∗*^ indicates the comparison with the control group, *P* < 0.05; ^#^ indicates the comparison with the spleen-kidney yang deficiency group, *P* < 0.05.

**Figure 2:** Comparison of Th17-related cytokine expression level in different groups ($\bar{x}$ ± *s*, pg/ml). The IL-6 expression levels of the control group, the damp-heat internal accumulation group, and the spleen-kidney yang deficiency group were (104.95 ± 40.95) pg/ml, (289.32 ± 84.26) pg/ml, and (192.28) ± 92.13) pg/ml, respectively; the IL-17 expression levels were (6.98 ± 2.25) pg/ml, (17.56 ± 3.02) pg/ml, and (15.21 ± 2.78) pg/ml, respectively; the IL-22 expression levels were (20.78) ± 9.42) pg/ml, (51.26 ± 12.41) pg/ml, (39.23 ± 9.36) pg/ml, respectively; the TNF-*α* expression levels were (10.13 ± 1.61) pg/ml, (28.45 ± 1.95) pg/ml, and (20.96 ± 1.35) pg/ml, respectively. ^*∗*^ indicates the comparison with the control group, *P* < 0.05; ^#^indicates the comparison with the spleen-kidney yang deficiency group, *P* < 0.05.

**Figure 3:** Comparison of Treg-related cytokine expression level in different groups ($\bar{x}$ ± *s*). (a) IL-10 expression level and (b) TGF-*β* expression level. Among them, the IL-10 expression levels of the control group, the damp-heat internal accumulation group, and the spleen-kidney yang deficiency group were (29.98 ± 9.89) ng/ml, (14.35 ± 3.95) ng/ml, and (18.32 ± 3.78) ng/ml, respectively; the TGF-*β* expression levels were (1268.58 ± 172.36) pg/ml, (932.56 ± 203.16) pg/ml, and (1006.35 ± 186.63) pg/ml, respectively. ^*∗*^ indicates the comparison with the control group, *P* < 0.05; ^#^ indicates the comparison with the spleen-kidney yang deficiency group, *P* < 0.05.

**Figure 4:** Comparison of Th17 and Treg cell ratios and Th17/Treg ratio in peripheral blood between the active UC groups ($\bar{x}$ ± *s*). (a) Th17 and Treg cell ratios in peripheral blood between the active UC groups and (b) Th17/Treg ratio in peripheral blood between the active UC groups. Among them, the Th17 cells ratios in the lightly active period group, the moderately active period group, and the severely active period group were (7.48 ± 2.35)%, (8.18 ± 2.45)%, (9.88 ± 2.02)%, respectively; the Treg cells ratios were (0.85 ± 0.23)%, (0.71 ± 0.18)%, (0.18 ± 0.20)%, respectively; the Th17/Treg ratios were (9.09 ± 2.98), (11.12 ± 3.26), (12.36 ± 3.66), respectively. ^*∗*^ indicates the comparison with the lightly active period group, *P* < 0.05; ^#^ indicates the comparison with the moderately active period group, *P* < 0.05.

**Figure 5:** The relationship between the proportion of Th17, Treg cells in the peripheral blood, and the ratio of Th17/Treg and the condition of UC patients. (a) Scatter plot of the correlation between the Th17 cell ratio and the Mayo scores, (b) scatter plot of the correlation between the Treg cell ratio and the Mayo scores, and (c) scatter plot of the correlation between the Th17/Treg ratio and the Mayo scores.

## Data Availability

The primary data to support the results of this study are available at reasonable request to the corresponding author.
